This article has been retracted.

# The Association between the Risk of Esophageal Cancer and Type 2 Diabetes Mellitus: An Updated Meta-Analysis

**DOI:** 10.1155/2022/8129771

**Published:** 2022-10-13

**Authors:** Runquan Zhou, Chenglu Huang, Zhilin Luo, Tianhu Wang

**Affiliations:** ^1^Department Of Thoracic Surgery, The Third Affiliated Hospital of Chongqing Medical University, Chongqing 401120, China; ^2^Department of Thoracic Surgery, Chongqing University Cancer Hospital, No. 181 Hanyu Road, Shapingba District, Chongqing 400030, China

## Abstract

**Background:**

A large amount of publications had reported the association between incidence of esophageal cancer (EC) and type 2 diabetes mellitus (T2DM) in the past decade. However, those papers' results are inconsistent on relationships between T2DM the incidence of EC. Therefore, the objective of this meta-analysis was to determine the relationship between T2DM and the risk of EC (including 2 histological types, esophageal adenocarcinoma [EADC] and esophageal squamous cell carcinoma [ESCC]).

**Method:**

We finally extracted 19 articles though Pubmed, Embased, and Cochrane library. Those identify extraction date including 14,312 cases and 24,959,067 control records and then mixed the relative risks (RRs) and corresponding 95% confidence intervals (95%CIs) through STATA.

**Results:**

We observed that there are significantly positive correlation between T2DM and EC risk (*RR* = 1.28, 95% CI: 1.05-1.57, *P* = 0.015).Also, our study showed positive correlation between T2DM and EADC (esophageal adenocarcinoma) risk (*RR* = 1.28, 95% CI: 1.05-1.57, *P* < 0.001). What's more, subgroup analysis based on ethnicity represented the Caucasian is more susceptible to EC (*RR* = 1.28 ,95% CI: 1.10-1.49, *P* = 0.001).

**Conclusion:**

Those results offer a recent epidemiological and integrated evidence to ascertain the correlations between T2DM and incidence of EC. Those results take public health implications on preventing T2DM and then depress the occurrence of EC. Our study also provides referenced information for the prevention. However, some data is still insufficient, and more research should be carried out.

## 1. Introduction

Esophageal cancer has become the commonest cancer around the world in the top eight and the cause of sixth cancer-related mortality, with the five-year survival ratio is not even close 20% [1, 2]. There are more than 570,000 new EC cases worldwide in 2018 [2]. In 2017, there were 234,624 new EC cases in China, mainly concentrated in Yanting County, Linxian County, North China (largely in the Taihang Mountains Area), and Central China (largely in the Dabie Mountains Area). It is reported that 212,586 people died from the EC every year [3]. Although there are surgery, chemotherapy, anti-immunotherapy and other comprehensive treatment, the prognosis of esophageal cancer is still not optimistic. According to pathological types, EC is classified into esophageal adenocarcinoma (EADC) and esophageal squamous cell carcinoma (ESCC). Acknowledged risk factors of ESCC include smoking, alcohol, mutation of enzymes' genes, achalasia of the cardia, corrosive trauma esophagus and hot drinks, chest radiation exposure, low socioeconomic status, poor state of mouth hygiene, and nutritional deficiencies [4, 5]. Poor intake of vegetables and fruits, selenium, zinc, and vitamin E deficiency were covered in other risk factors. Interestingly, the protective factor is high BMI [4–17]. Acknowledged risk factors for EADC include Barrett's esophagus, symptomatic gastro-esophageal reflux disease (GERD), visceral obesity, smoking, drugs that relaxes the low esophageal sphincter, high BMI, as well as a poor intake of vegetables and fruit and high intake of processed meat [18, 19]. For achieving a great progress in the prognosis of EC, it is necessary to investigate and develop preventive measures.

More and more studies represent type 2 diabetes mellitus (T2DM) could increase incidence of gastroenteric tumors now, like liver cancer and pancreatic cancer [20–23]. In particular, the incidence of those gastroenteric tumors is higher in the old or the male [23]. At present, most studies have studied the relationship between incidence of EC and T2DM, but there is no exact data to explain the relationship between incidence of EC and T2DM. Some meta-analyses suggested that T2DM would increase the incidence of EC. While the correlations between T2DM and the risk of EC (including EADC or/and ESCC) were seldomly performed in those studies. What's more, those studies had been seldomly investigating the individual effect of each T2DM individual in EC (including EADC or/and ESCC) comprehensively. So our aim was to perform a meta-analysis to confirm risk of EC (including EC's subtypes ESCC and EADC) in T2DM and nondiabetic individual.

## 2. Material and Method

### 2.1. Literature Search

All English literatures were searched from Pubmed, Embase, and Cochrane (June 1994 to October 2020) by searching for terms, with the following text word or Medical Subject Heading (MeSH) terms in the title or abstract: “{esophagus} OR {esophageal} OR {oesophagus} OR {oesophageal}” AND“{cancer} OR {carcinoma} OR {adenocarcinoma} OR {squamous cell carcinoma} OR {tumor} OR {malignant} OR {malignancy} OR {neoplasm} OR {neoplasia} OR {oncology}” AND“{diabetes mellitus} OR {diabetes complications}” AND“{diabet}” AND“{ IDDM} OR { NIDDM} OR {MODY} OR {T1DM} OR {T2DM } OR {T1D} OR {T2D}” AND“{inculin^∗^} OR {noninsulin^∗^}” AND“{depend^∗^}“AND “{odds ratio} OR {OR} OR {hazard risk} OR {hazard ratio} OR {HR} OR {relative risk} OR {RR} OR {rate ratio} OR {P} OR {P value} OR {P=} OR {association} OR {associated} OR {confidence interval} OR {CI} OR {censor} OR {Kaplan-Meier} OR {Cox model} OR {Proportional hazard model} OR {log-rank}.” We selected those publications by screening their title, abstract, and even full article if necessary.

### 2.2. Criteria for Inclusion

We comply with following criteria to select publications/literatures: (1) The exposure factor was T2DM (or contains T2DM); (2) the prognostic indicator are the risk of EC or its subtypes; (3) studies were all written in English; and (4) provide relative risk (RR) estimates and their 95% confidence intervals (95% CI), or report raw data from which the RR and 95% CI can be calculated. The exclusion criteria are as follows: (1) no or insufficient information is available to calculate the relevant estimates; (2) the outcome indicator was cancer mortality or survival rate (not incidence). (3) patients diagnosed with T1DM (We found that the association between EC and type 1 diabetes was not mentioned in almost of the literature; therefore, the relation between type 1 diabetes and EC was not necessary in this meta-analysis.).

### 2.3. Literature Selection and Assessment

We (Dr. Zhou. and Dr. Huang) selected and assessed literatures (according to Jadad Quality Assessment Scale) independently, and any discrepancies were resolved by consensus. Jadad quality assessment rating scale can be divided into 2 level. The scale range between 0 to 3 is considered as a low quality research. On the contrary, the scale range between 0 to 3 is considered as a high quality research. In addition, ethnicity was classified into Asian and Caucasian.

### 2.4. Data Extraction

Two investigators (Dr. Zhou. and Dr. Huang) collected following relevant date from included literatures separately: author, publish time, country/region, ethnicity, study design, assessment method, comparison of population, source/study population, cancer type, controls/cohort size, follow-up years, risk factors, relevant estimate type (odds ratio (OR), RR, hazard ratio (HR), and 95% CI), and the adjustment variables. Finally, Dr. Luo and Dr. Wang checked all data. If we get a disagreement, we will solve it by further discussion.

### 2.5. Statistical Analysis

All extracted data from included literatures meta-analysis processed by STATA 16.0. Also, all extracted data was regarded as a binary variable. The association between incidence of EC and T2DM were evaluated by RRs and 95% CIs by random-effects models. Heterogeneity among studies was evaluated by Cochran's Q test and *I*^2^ values [24, 25]. *I*^2^ is divided this meta-analysis results into three grades: ≤25%, 25-50%, and ≥50 (heterogeneity was low, medium, and large, respectively). The stability of the results was evaluated by the sensitivity analysis so that we can try to explain heterogeneity. The publication bias of each study was assessed by Egger's test. When *P* < 0.05, we decide to think the difference was statistically significant.

## 3. Result

We searched the initial total 1566 literatures through Pubmed, Embase, and Cochrane. We finally screen out total 19 literatures [26–44] after a strict and cautious review (Figure 1). As presented in Table 1, those studies include 14312 cases and 24959067 controls. In terms of esophageal cancer histological type, 3 studies [26, 40, 41] were performed in ESCC and 7 studies [29, 34, 37, 40–42, 44] in EADC, and 11 [27, 28, 30–33, 35, 36, 38, 39, 43] studies did not instruct type of EC. For study design, 5 studies [28, 33, 34, 36, 40] were performed in a cohort study and 14 [26, 27, 29–32, 35, 37–39, 41–44] studies in a case-control study. To ethnicity, 4 studies [31, 32, 35, 38] were performed in Asians and 10 studies [26–28, 30, 33, 36, 39–41, 43] in Caucasians, and 5 studies [29, 34, 37, 42, 44] did not instruct specific number of ethnicity.

As presented in meta-analysis, a significant association was found between T2DM and risk of EC (*RR* = 1.28, 95%*CI* = 1.05–1.57, *I*^2^ = 96.9%, Figure 2) and was presented based on 19 studies. Because of significant heterogeneity (*I*^2^ = 96.9%, *P* < 0.001), we analyze the all data in random-effects models.

When we concentrated on the 7 studies [29, 34, 37, 40–42, 44] specified for the subtypes of EADC, we noticed a significant association between risk of EADC and T2DM (*RR* = 1.22, 95% CI: 1.38–1.55, *P* < .001, Figure 3). We also limited the meta-analysis to the 10 studies [26–28, 30, 33, 36, 39–41, 43] specified for the subtypes of Caucasians, founding that Caucasians were more likely to develop esophageal cancer (*RR* = 1.28, 95% CI: 1.10-1.49, *P* = 0.001, Figure 4).

Moreover, we decided to adopt Begg funnel chart and Egger's test to test the potential publication bias. We found no statistic significant publication bias in our main study (T2DM and EC risk) (Begg correlation test (*P* = 0.726) and Egger test (*P* = 0.479), Figure 5). There were few evidences of potential publication bias for the association between T2DM and risk of EC. Subsequently, the funnel plots based on Caucasians showed that there was hardly any publication bias (Begg correlation test (*P* = 0.806) and Egger test (*P* = 0.573), Figure 6). And the funnel plots based on EADC revealed that there was no publication bias (Begg correlation test (*P* = 0.536) and Egger test (*P* = 0.731), Figure 7).

## 4. Discussion

Recently, more and more researches have reported the association between T2DM and tumor. However, those results rarely refer to EC and inconsistent. Our research suggested that T2DM may increase the incidence of EC, especially EADC. Our subgroup analysis suggested by ethnicity suggested that Caucasians may be a risk factor; Caucasians are more susceptible to EC.

T2DM may be linked to EC through long-term high glucose levels in blood [45–48] and metabolic syndrome (including insulin resistance) [49–51]. From histological type, EC can be classified by EADC and ESCC. On the one hand, T2DM caused gastroesophageal abnormalities which can lead to GERD. GRED promotes the occurrence of EADC. Smoking, alcohol consumption, and low BMI are recognized risk factors for ESCC [34, 52–54]. On the other hand, obesity and high BMI, common in diabetes, were risk factors for EADC and protective factors for ESCC [55, 56], while hyperinsulinemia is related to the increase of bioactive serum IGF-1, which can also promote the development of EADC [57–60]. T2DM will cause patients hyperinsulinemia, which will increase risk of EC by adjusting serum levels of IGF1.The hyperinsulinemia results in a constant increase in serum insulin levels among T2DM patients, which decreases the levels of growth factor binding protein 1(IGFBR 1) and IGFBP 2.Those effects lead to the rise of IGF1 in blood, which increases risk of EC [61]. The expression of the isoform (IR-A) is predominant in many malignant cells.T2DM patients cells with high levels of insulin receptor (IR) content, which will bind to IR-A. Then, it will result in more caryomitosis than metabolic effects and promoting the growth of cancer consequently [62, 63]. These were a large of research has suggested the use of metformin could reduce cancer risk of occurrence in T2DM patients [64, 65]. The mechanism of anticarcinogenic may attribute to that the metformin prompt release of Adenosine 5′-monophosphate– (AMP–) activated protein kinase (AMPK) so that it can inhibit of tumor cellular protein's synthesis and increase, with low level of insulin [66, 67]. However, the use of antidiabetic drugs has not been proved to reduce the incidence of EC.

Significant heterogeneities were found in our result. Hence, sensitivity analysis was performed to assess the stability of the results. After sensitivity analysis, the three articles were found to have great heterogeneity. In J. L. Dixon's study [34], the control group was not the traditional recognized healthy people like other studies, but people had been diagnosed with GERD and treated with fundoplication within a year; furthermore, 124 female patients were excluded. The symptoms of early EC were not obvious and were usually diagnosed in the late stage. However, in Abureesh's study [28], the subjects were 20-50 years old EC patients, so the number of esophageal cancer patients in the study was not completely accurate. Also, T2DM was not easily found in young people, so the number of diabetes was not accurate neither. In Roy G.P.J. de Jong's study [33], people with T2DM who have not been treated by antidiabetic drug or whose diabetes has not been detected may also be included in the health population. The control group may get any diseases other than T2DM or the exclusion criteria above. This can affect their survival and decrease their chances of cancer. In addition, tumor subgroups were classified by their anatomical location, and there was no exclusion criterion. Tumors in the esophageal location were not identified as primary esophageal cancer, so there was a large difference. In general, what leads to the heterogeneity of this meta-analysis is different exposure, outcome, and other indicators defined by different studies.

### 4.1. Limitation

The limitations of our study as follow: (1) some study still missed by our comprehensive search. (2) Different studies list many different adjusted factors (such as sex, age, education, birth place, smoking, social statue, anti-mellitus drugs, and body mass index (BMI)) which may influence our meta-analysis results. (3) Trying to find out source of significant heterogeneities, we performed subgroup analysis. Unfortunately, only ethnicity could be responsible for parts of heterogeneity. (4) Included studies take different historical types as research subjects. So our result of ORs and 95% CI should be explained carefully.

## 5. Conclusion

Summarily, this study suggested that T2DM had positive association with a growing EC risk, especially EADC and between Caucasian. Hence, for T2DM patients, they should focus not only on treating diabetes, but also on early screening for cancer, especially like EC whose early symptoms hard to detect. Also, our study can provide some useful information for T2DM patients and help them help the implementation of the individualized therapeutic interventions in order to reduce the occurrence of EC risk. However, some data is still insufficient, and more well-designed prospective study should be carried out.

## Figures and Tables

**Figure 1:** Search strategy and study selection.

**Figure 2:** The forest plot of overall effect for association between T2DM and EC risk.

**Figure 3:** The forest plot of overall effect for association between T2DM and EADC risk.

**Figure 4:** The forest plot of overall effect for association between EC and Caucasian risk.

**Figure 5:** Funnel plot analysis of all included articles. Begg correlation test (*P* = 0.726) and Egger test (*P* = 0.479).

**Figure 6:** Funnel plot analysis of articles specified for the subtypes of Caucasians. Begg correlation test (*P* = 0.806) and Egger test (*P* = 0.573).

**Figure 7:** Funnel plot analysis of articles specified for the subtypes of EADC. Begg correlation test (*P* = 0.536) and Egger test (*P* = 0.731).

**Table 1:** The characteristics of including studies.

First author	Year	Country/region	Ethnicity	Study design	Assessment method	Source/study population	Cancer type	Follow-up years	Score of Jadad
La Vecchia, C	1994	Italy	Caucasian	Case-control study	Questionnaire	General hospitals in the Greater Milan area	EC	10 years	4
Yan Gong	2012	China	Asian	Case-control study	Patients whose fasting glucose was >7.8 mmol/L at least twice	Chinese PLA General Hospital	EC	4 years 10 months	4
J. L. Dixon	2015	USA	NA	Prospective cohort study	Questionnaire	Interrogation of an administrative database	EAC	1 year	5
Xuejuan Jiang	2012	USA	NA	Case-control study	Questionnaire	Los Angeles County Cancer Surveillance	EAC	NA	5
RE Neale	2009	Australia	Caucasian	Case-control study	Questionnaire	Major treatment centers and statebases cancer throughout mainland Australia	OAC	4 years	4
							GOJAC	4 years	
							OCSS	4 years	
Yang Hu	2014	USA	Caucasian	Prospective cohorts study	Questionnaire	The Nurses' Health Study (women) and the Health Professionals (man)	EC	26/36 years	5
Abureesh, Mohammad MD	2020	USA	NA	Prospective cohorts study	NA	Major US healthcare systems	EC	20years	4
Shih-wen Lin	2011	USA	Caucasian	Prospective cohorts study	Questionnaire	NIH-AARP	ESCC	7.96 years	6
							EADC	7.96 years	
J. H. RUBENSTEIN	2005	USA	NA	Case-control study	NA	United States Veterans Affairs (VA) National Patient Care Datasets (NPCD)	OAC	20 years	5
Sangeeta Agrawal	2014	USA	NA	Case-control study	Questionnaire	Dayton Veterans Affairs Medical Center database	OAC	20 years	5
Cristina Bosetti	2012	Italy and Switzerland	Caucasian	Case-control study	Questionnaire		ESCC	18 years	4
Claudia Becker	2013	UK	Caucasian	Case-control study	NA	The general practice research database in the UK	EC	16 years	6
Kao-chi Cheng	2012	China	Asian	Case-control study	NA	National Health Insurance (NHI) program in Taiwan	EC	9 years	5
KK Cheng	2000	UK	Caucasian	Case-control study	Interview	Regional Health Authorities (RHA) of East Anglia and Oxford, part of Trent RHA and Eastern Scotland	EC	2 years	4
Wen-Ko Chiou	2011	China	Asian	Case-control study	Examination	Chang Gung Memorial Hospital	EC	1.5 years	6
Kevin M. Reavis	2004	USA	NA	Case-control study	Questionnaire	Portland VA Medical Center	EAC	5 years	5
Marie-Claude Rousseau	2005	Canada	Caucasian	Case–control study	Questionnaire	Major hospitals in Montreal	EC	6 years	4
Kiyonori Kuriki	2007	Japen	Asian	Case–control study	Questionnaire	The Aichi Cancer Center Hospital (ACCH)	EC	12 years	4
Roy G.P.J. de Jong	2018	UK	Caucasian	Cohort study	UK Clinical Practice Research Datalink (CPRD)		EC	24 years	6

## Data Availability

All data and materials were obtained from Pubmed, Embase, and Cochrane. All data generated or analyzed during this study are included in this published article and its supplementary information files.

## Abbreviations

EC: Esophageal cancer
T2DM: Type2 diabetes mellitus
EADC: Esophageal adenocarcinoma
ESCC: Esophageal squamous cell carcinoma
RRs: Relative risks
CIs: Confidence intervals
GERD: Gastroesophageal reflux disease
OR: Odds ratio
HR: Hazard ratio
GFBP1: Growth factor binding protein 1
GFBP2: Growth factor binding protein 2
IR: Insulin receptor
(AMP): Adenosine 5′-monophosphate
AMPK: Activated protein kinase.
